The article "Statistical Analysis of the COVID-19 Mortality Rates with Probability Distributions: The Case of Pakistan and Afghanistan" was published in 2022. Journal: Comput Math Methods Med.

# Statistical Analysis of the COVID-19 Mortality Rates with Probability Distributions: The Case of Pakistan and Afghanistan

**DOI:** 10.1155/2022/4148801

**Published:** 2022-07-25

**Authors:** Javid Gani Dar, Muhammad Ijaz, Ibrahim M. Almanjahie, Muhammad Farooq, Mahmoud El-Morshedy

**Affiliations:** ^1^Department of Mathematical Sciences, IUST, Kashmir, India; ^2^Department of Mathematics and Statistics, The University of Haripur, Haripur, KPK, Pakistan; ^3^Department of Mathematics, College of Science, King Khalid University, Abha 62529, Saudi Arabia; ^4^Statistical Research and Studies Support Unit, King Khalid University, Abha 62529, Saudi Arabia; ^5^Department of Statistics, University of Peshawar, KPK, Pakistan; ^6^Department of Mathematics, College of Science and Humanities in Al-Kharj, Prince Sattam bin Abdulaziz University, Al-Kharj 11942, Saudi Arabia; ^7^Department of Mathematics, Faculty of Science, Mansoura University, Mansoura 35516, Egypt

## Abstract

The COVID-19 pandemic has shocked nations due to its exponential death rates in various countries. According to the United Nations (UN), in Russia, there were 895, in Mexico 303, in Indonesia 77, in Ukraine 317, and in Romania 252, and in Pakistan, 54 new deaths were recorded on the 5th of October 2021 in the period of months. Hence, it is essential to study the future waves of this virus so that some preventive measures can be adopted. In statistics, under uncertainty, there is a possibility to use probability models that leads to defining future pattern of deaths caused by COVID-19. Based on probability models, many research studies have been conducted to model the future trend of a particular disease and explore the effect of possible treatments (as in the case of coronavirus, the effect of Pfizer, Sinopharm, CanSino, Sinovac, and Sputnik) towards a specific disease. In this paper, varieties of probability models have been applied to model the COVID-19 death rate more effectively than the other models. Among others, exponentiated flexible exponential Weibull (EFEW) distribution is pointed out as the best fitted model. Various statistical properties have been presented in addition to real-life applications by using the total deaths of the COVID-19 outbreak (in millions) in Pakistan and Afghanistan. It has been verified that EFEW leads to a better decision rather than other existing lifetime models, including FEW, W, EW, E, AIFW, and GAPW distributions.

## 1. Introduction

The first case of COVID-19 infection was located in Pakistan on February 26, 2020, in Karachi—a recent returnee from Iran. From that point onward, the spread of contaminations sped up, and on March 18, 2020, it was affirmed that the infection had spread to all regions of Pakistan. More than a hundred deaths apart from more than six thousand infected people were reported in the first seven weeks of this outbreak [1]. Pakistan has the third-highest number of cases in South Asia after India and Bangladesh, while it stands 7th in Asia as of September 16, 2021, with a 26th position worldwide. The first death was reported on March 20 in Sindh province, and the community transmission was spread rapidly all over the country.

In a country like Pakistan, the graph started to follow an upward trajectory in March 2020 and peaked in June when it slowly started to decline and flattened in August and September. But again, it started to increase in October of the same year, reflecting the bathtub shape in the data. Figures 1(a) and 1(b) show the average infection rates.

Many researchers have conducted various studies to investigate the COVID-19 outbreak, such as Singh et al. who explored how to predict the COVID-19 pandemic for the top 15 countries using the ARIMA model [2]. The worldwide death rates were estimated by Chaurasia and Pal, by employing the ARIMA and regression models [3]. Chakraborty and Ghosh utilized a regression tree and ARIMA model to forecast the short time of COVID-19 cases in multiple countries and the risk of COVID-19 by finding various demographic characteristics beside some disease characteristics within these countries [4]. Yousaf et al. [5] utilized the autoregressive integrated moving average (ARIMA) model to predict infections, deaths, and recoveries. Fong et al. [6] considered small data for early forecasting, while Petropoulos and Makridakis [7] also applied the forecasting model. Chen et al. [8] designed an algorithm for predicting COVID-19 data, while Nayak et al. [9] and Wolkewitz et al. [10] applied a probabilistic model to analyze COVID-19 data. The size of the COVID-19 epidemic has been worked out by Yue et al. [11] with the help of surveillance systems, and a similar study to estimate the final size of the COVID-19 epidemic has also been discussed by Syed and Sibgatullah [12]. Mizumoto et al. [13] estimated the asymptomatic proportion of COVID-19. Many researchers applied various statistical models to predict data analysis. For example, Sukhanova et al. [14] forecast the macroeconomic indices with the help of ARIMA, vector autoregression (VAR), and simultaneous equation system. Yu et al. [15] predict the tourism demand by utilizing the SARIMA model and neural network (NN). To examine the accuracy with which long-term scenarios can be predicted in patients with coronary artery disease, Lee et al. [16] applied Cox regression. The results showed that model-based prediction was considered better as compared to doctors' prediction.

Many lifetime distributions are available in the literature to predict the COVID-19 data, but these distributions are unable to model the data more precisely. For example, the Weibull (W) distribution introduced by Weibull [17] and the exponential (Ex) distribution by Epstein [18] along with other lifetime distributions are unable to model the COVID-19 data or any other data related to any infections of the disease that does not follow a constant rate (monotonic data). In daily life situations, the data does not always follow a monotonic failure function; rather, it follows a nonmonotonic failure function. For example, patients with tuberculosis have a higher risk in the early stages but a lower risk later on. A similar form of nonmonotonicity occurs in infants because the hazards for infants are highest in the early stages and gradually reduce as they develop, but the danger increases again as they become older, resulting in the bathtub shape. The researchers are trying to introduce functions that are more flexible as well as and can capture the nonmonotonic hazard rate functions. For example, Cordeiro et al. [19], El-Gohary et al. [20], Ijaz et al. [21], and Farooq et al. [22] worked on introducing the new distributions. We recommend recent research studies: Ijaz et al. [21, 23] and Ijaz et al. [24].

In practice, the modeling of real phonon becomes more complex when the number of unknown's parameters is large. There are two main significant advantages of the probability models in this paper. First, it presents a best fitted model which is more flexible with fewer unknown parameters. Secondly, it leads us to better results for various hazard rate shapes, particularly in a bathtub shape where the curves are flatted at the middle and skewed on either side. Note that the distribution in this paper may not be considered as a best fitted model for the data sets with extreme values or even when there is an outlier.

## 2. Material and Methodology

The current research study focuses on the best fitted probability model which has more parameters as compared to some existing models. In this paper, the best fitted model has increased a shape parameter (*d*) in the family of distributions introduced by [22]. The CDF and PDF of the proposed probability model take the following forms:

(1) $$\begin{array}{c} F\left(x\right)={\left(\frac{e^{aF\left(x\right)}-1}{e^{a}-1}\right)}^{d},\;x\text{ and }a,\;d>0, \end{array}$$

(2) $$\begin{array}{c} f\left(x\right)=\frac{adf\left(x\right)e^{aF\left(x\right)}{\left(e^{aF\left(x\right)}-1\right)}^{d-1}}{{\left(e^{a}-1\right)}^{d}}. \end{array}$$

By putting the CDF and PDF of the Weibull distribution, Equations (1) and (2) take the following form:

(3) $$\begin{array}{c} F\left(x\right)={\left(\frac{\left(e^{a\left(1-e^{-{bx}^{c}}\right)}-1\right)}{e^{a}-1}\right)}^{d},\;x>0,\;a,\;b,\;c,\text{ and }d>0, \end{array}$$

(4) $$\begin{array}{c} f\left(x\right)=\frac{{abcdx}^{c-1}e^{a\left(1-e^{-{bx}^{c}}\right)-{bx}^{c}}{\left(e^{a\left(1-e^{-{bx}^{c}}\right)}-1\right)}^{d-1}}{{\left(e^{a}-1\right)}^{d}}, \end{array}$$

where “*b*” is the scale and “*c*” and “*d*” are the shape parameters.

Figure 2 defines the shapes of the CDF and PDF described in (3) and (4), respectively.

### 2.1. The Survival *S*(*x*) and Hazard *h*(*x*) Rate Function

By definition, *S*(*x*) and *h*(*x*) functions are, respectively, defined by

(5) $$\begin{array}{c} S\left(x\right)=1-F\left(x\right),\\ h\left(x\right)=\frac{f\left(x\right)}{S\left(x\right)}. \end{array}$$

Using (3) and (4), we get

(6) $$\begin{array}{c} S\left(x\right)=\frac{{\left(e^{a}-1\right)}^{d}-{\left(e^{a\left(1-e^{-{bx}^{c}}\right)}-1\right)}^{d}}{{\left(e^{a}-1\right)}^{d}},\\ h\left(x\right)=\frac{{abcdx}^{c-1}e^{a\left(1-e^{-{bx}^{c}}\right)-{bx}^{c}}{\left(e^{a\left(1-e^{-{bx}^{c}}\right)}-1\right)}^{d-1}}{{\left(e^{a}-1\right)}^{d}-{\left(e^{a\left(1-e^{-{bx}^{c}}\right)}-1\right)}^{d}}. \end{array}$$

Figure 3 defines various shapes of the hazard rate function.

## 3. Statistical Properties

### 3.1. Quantile Function

The quantile function is defined by

(7) $$\begin{array}{c} p\left(X\leq x\right)=q. \end{array}$$

Using (3), we get

(8) $$\begin{array}{c} \left(e^{a\left(1-e^{-{bx}^{c}}\right)}-1\right)=q^{1/d}\left(e^{a}-1\right). \end{array}$$

The final result for *X* can be obtained as

(9) $$\begin{array}{c} x={\left(\frac{-1}{b}\log\left(\frac{a-\log\left(1+q^{1/d}\left(e^{a}-1\right)\right)}{a}\right)\right)}^{1/c}, \end{array}$$

where *q* ~ *U*[0, 1].

### 3.2. *r*th Moment

The *r*th moment can be obtained by

(10) $$\begin{array}{c} E\left(x^{r}\right)=\int x^{r}f\left(x\right)dx,\\ E\left(x^{r}\right)=\int_{0}^{\infty }\frac{x^{r}{abcdx}^{c-1}e^{a\left(1-e^{-{bx}^{c}}\right)-{bx}^{c}}{\left(e^{a\left(1-e^{-{bx}^{c}}\right)}-1\right)}^{d-1}dx}{{\left(e^{a}-1\right)}^{d}}. \end{array}$$

Using *z* = *e*^*a*(1 − *e*^−*bx*^*c*^^)^, then *dz* = *abcx*^*c*−1^*e*^*a*(1 − *e*^−*bx*^*c*^^)−*bx*^*c*^^*dx* and *x* = (−1/*b*log(1 − log*z*/*a*))^1/*c*^.

(11) $$\begin{array}{c} E\left(x^{r}\right)=\frac{d{\left(-1/b\right)}^{r/c}}{{\left(e^{a}-1\right)}^{d}}\int_{1}^{e^{a}}{\left(\log\left(1-\frac{\log z}{a}\right)\right)}^{r/c}{\left(z-1\right)}^{d-1}dz. \end{array}$$

Using (log(1 − log*z*/*a*))^*r*/*c*^ = ∑_*k*=1_^∞^(−1)^*k*+*r*/*c*^(*k*)^*c*/*r*^(−log*z*/*a*)^*kr*/*c*^ for |*l*og*x*/*a*| < 1 and ${\left(z-1\right)}^{d-1}=\sum_{n=0}^{\infty }{\left(-1\right)}^{1+d+n}\left(\begin{array}{c} d-1\\ n \end{array}\right)z^{n}$,

finally, we obtained

(12) $$\begin{array}{c} =\frac{d{\left(-1/b\right)}^{r/c}}{{\left(e^{a}-1\right)}^{d}}\overset{\infty }{\underset{k=1}{\sum }}\overset{\infty }{\underset{n=0}{\sum }}{\left(-1\right)}^{k+r/c}{\left(-1\right)}^{1+d+n}{\left(k\right)}^{c/r}\left(\begin{array}{c} d-1\\ n \end{array}\right)\frac{\left[{\left(-1\right)}^{kr/c}{\left\{-\left(n+1\right)a\right\}}^{-kr/c}\Gamma \left(kr/c+1,-\left(n+1\right)\log a\right)\right]}{n+1}. \end{array}$$

### 3.3. Order Statistics

The *i*^th^ order statistic of the PDF is given by

(13) $$\begin{array}{c} f\left(i,n\right)\left(x\right)=\frac{n!}{\left(i-1\right)!\left(n-i\right)!}f\left(x\right)F{\left(x\right)}^{i-1}{\left(1-F\left(x\right)\right)}^{n-i}. \end{array}$$

Letting Equations (3) and (4), the 1^st^ and *n*^th^ order statistics of EFEW can be obtained, respectively, by using *i* = 1 and  *i* = *n* as

(14) $$\begin{array}{c} f\left(1,n\right)=\frac{{nabcdx}^{c-1}e^{a\left(1-e^{-{bx}^{c}}\right)-{bx}^{c}}{\left(e^{a\left(1-e^{-{bx}^{c}}\right)}-1\right)}^{d-1}{\left(e^{a}-e^{a\left(1-e^{-{bx}^{c}}\right)}\right)}^{\left(n-1\right)d}}{{\left(e^{a}-1\right)}^{nd}},\\ f\left(n,n\right)=\frac{{nabcdx}^{c-1}e^{a\left(1-e^{-{bx}^{c}}\right)-{bx}^{c}}{\left(e^{a\left(1-e^{-{bx}^{c}}\right)}-1\right)}^{nd-1}}{{\left(e^{a}-1\right)}^{nd}}. \end{array}$$

### 3.4. Skewness and Kurtosis

The mathematical form of the skewness and kurtosis is given below:

(15) $$\begin{array}{c} S=\frac{Q\left(6/8\right)+Q\left(2/8\right)-2Q\left(4/8\right)}{Q\left(6/8\right)-Q\left(2/8\right)},\\ K=\frac{Q\left(7/8\right)+Q\left(3/8\right)-Q\left(5/8\right)-Q\left(1/8\right)}{Q\left(6/8\right)-Q\left(2/8\right)}, \end{array}$$

where *α*^ln(1 − e^−*by*^)^log(*α*)*β*/(1 − *α*^ln(1 − e^−*by*^)^)(e^*by*^ − 1) describes quartile values.

Table 1 clearly shows that EFEW can model the normal, positively skewed data, or even the data skewed to the left.

## 4. Special Cases

The special cases of EFEW are as follows.

**Case 1 . When *d* = 1.**

By putting *d* = 1 in (3) and (4), we derive the CDF and PDF of the flexible exponential Weibull (FEW) distribution. The mathematical form is described as

(16) $$\begin{array}{c} F\left(x\right)=\frac{e^{a\left(1-e^{-{bx}^{c}}\right)}-1}{e^{a}-1},\;x>0,\;b>0,\;c>0,\text{ and }a\neq 1,\\ f\left(x\right)=\frac{{abcx}^{c-1}e^{a\left(1-e^{-{bx}^{c}}\right)-{bx}^{c}}}{e^{a}-1}. \end{array}$$

**Case 2 . When *d* = 1 and *c* = 1.**

Putting *d* = 1and *c* = 1 in (3) and (4) shall refer to the CDF and PDF of the gull alpha power exponential distribution (GAPE). The mathematical form is described as

(17) $$\begin{array}{c} F\left(x\right)=\frac{e^{a\left(1-e^{-bx}\right)}-1}{e^{a}-1},\;x>0,\;b>0,\text{ and }a\neq 1,\\ f\left(x\right)=\frac{{abe}^{a\left(1-e^{-bx}\right)-bx}}{e^{a}-1}. \end{array}$$

**Case 3 . When *d* = 1 and *c* = 2.**

If we replace *d* = 1 and *c* = 2 in (3) and (4), the CDF and PDF will become NF Rayleigh (NFPR) distribution. Mathematically, the CDF and PDF of NFPR are

(18) $$\begin{array}{c} F\left(x\right)=\frac{e^{a\left(1-e^{-{bx}^{2}}\right)}-1}{e^{a}-1},\;x>0,\;b>0,\text{ and }a\neq 1,\\ f\left(x\right)=\frac{{abcxe}^{a\left(1-e^{-{bx}^{2}}\right)-{bx}^{2}}}{e^{a}-1}. \end{array}$$

## 5. Parameter Estimation

The log likelihood function of Equation (4) is defined by

(19) $$\begin{array}{c} \log\left(L\right)=n\log\left(\frac{abcd}{{\left(e^{a}-1\right)}^{d}}\right)+\left(c-1\right)\sum \log x_{i}+a\sum \left(1-e^{-{bx}^{c}}\right)-\sum {bx}^{c}+a\left(d-1\right)\sum \left(1-e^{-{bx}^{c}}\right). \end{array}$$

The partial derivatives of (19) with respect to parameters are obtained by

(20) $$\begin{array}{c} \frac{d}{d\left(a\right)}\log\left(L\right)=\left(d-1\right)\left(-nd\log\left(e^{a}-1\right)-e^{-{bx}^{c}}+1\right)-\frac{\left(d-1\right){ande}^{a}}{e^{a}-1}+\frac{n}{a}-e^{-{bx}^{c}}+1,\\ \frac{d}{d\left(b\right)}\log\left(L\right)=a\left(d-1\right)\sum x^{c}e^{-b\sum x^{c}}+a\sum x^{c}e^{-b\sum x^{c}}+\frac{n}{b}-\sum x^{c},\\ \frac{d}{d\left(c\right)}\log\left(L\right)=\frac{-e^{-b\sum x^{c}}\left(\left(\left(b\sum x^{c}\log\left(x\right)-\sum \log\left(x\right)\right)c-n\right)e^{\sum {bx}^{c}}-abcd\sum x^{c}\log\left(x\right)\right)}{c},\\ \frac{d}{d\left(d\right)}\log\left(L\right)=a\left(-\log\left(e^{a}-1\right)nd-e^{-b\sum x^{c}}+1\right)-a\log\left(e^{a}-1\right)n\left(d-1\right)+\frac{n}{d}. \end{array}$$

The above expressions are not in closed form, but still, the numerical solution is possible by using various mathematical techniques.

## 6. Applications

In this section, the COVID-19 death data of Pakistan and Afghanistan were considered to delineate the real-life applications by means of AIC, CAIC, BIC, and HQIC.

It should be noted that the model with a fewer value of these criteria is considered as the best model among others.

The data sets with the URL https://github.com/owid/covid-19-data are taken from May 2, 2020, till July 4, 2021, for Pakistan and Afghanistan. Tables 2 and 3 respectively defines the mortality rates in Pakistan and Afghanistan.

In Figure 4, both the theoretical and empirical graphs depict that the EFEW is the best fitted line as compared to other existing distributions and can be justified from Tables 4 and 5.

Figure 5 demonstrates the Q-Q and P-P plot of the COVID-19 death data. The Q-Q plot demonstrates that most of the data points, except a few points on the upper tail, follow a linear pattern on the line, while the P-P plot also indicates a reasonably good fit and indicates that the EFEW reasonably describes the empirical data distribution along with empirical and theoretical densities and their CDF.

Figure 6 depicts the pattern of the hazard rate function. The curve clearly crosses the diagonal line, and hence, the data follows a nonmonotonic hazard rate function.

Table 4 shows the Cramer-Mises (W) and Anderson-Darling (A) maximum likelihood estimates, standard errors, and log-likelihood values.  Table 5 shows the best model selection criterion. The results of Tables 5 and 6 depict the smaller values for FEW among others using this goodness of fit criteria and hence show that EFEW provides a flexible fit over exponential (E), Weibull (W), Exponential-Weibull (Ex-W), Algoharai inverse flexible Weibull (AIFW), and gull alpha power Weibull (GAPW) distributions.

Figure 7 shows the theoretical and empirical PDF and CDF of EFEW distribution using the COVID-19 death data from Afghanistan. Both the theoretical and empirical graphs clearly depict that the EFEW is the best fitted line as compared to other existing distributions and can be justified from the numerical values presented in Tables 6 and 7.

Figure 8 demonstrates the Q-Q and P-P plot of the COVID-19 death data from Afghanistan. The Q-Q plot demonstrates that most of the data points, except a few points on the upper tail, follow a linear pattern on the line, while the P-P plot also indicates a reasonably good fit and indicates that the EFEW reasonably describes the empirical data distribution along with empirical and theoretical densities and their CDF.

Figure 9 follows the same pattern as Figure 6 which means that the death rate in Afghanistan also follows a nonmonotonic shape.

The results of Tables 6 and 7 show that by employing these criteria, smaller values are achieved for EFEW, and hence, EFEW gives a flexible fit over FEW, E, W, Ex-W, AIFW, and GAPW.

## 7. Simulation Study of EFEW Distribution

A simulation study has been performed to check the consistency of the parameters of the EFEW distribution. We consider two set of parameter values, i.e., *a* = 0.5, *b* = 0.05, *c* = 1.5, and *d* = 0.5 and *a* = 0.6, *b* = 0.05, *c* = 1.77, and *d* = 0.6. A simulation is performed with 1000 replications. A sample of sizes *n* = 40, 70, 100, 150 and *n* = 100, 200, 300, 400 are drawn, respectively, and the bias and mean square error (MSE) are estimated. The mathematical forms are described as

(21) $$\begin{array}{c} \text{MSE}=\frac{1}{W}\overset{W}{\underset{i=1}{\sum }}{\left(\overset{\wedge }{\alpha_{i}}-\alpha \right)}^{2},\\ \text{Bias}=\frac{1}{W}\overset{W}{\underset{i=1}{\sum }}\left(\hat{\alpha_{i}}-\alpha \right). \end{array}$$

Table 8 defines the average mean square errors and biases of each parameter using small and large sample sizes taken from EFEW. It is quantified that when we increase the sample of size *n*, the average values of mean square errors and bias decrease with different values of parameters.

## 8. Conclusion

In this article, the best fitted model (EFEW) is pointed out for modeling the death rates of coronavirus. Various statistical properties of the proposed model have been discussed. The significance of EFEW has been evaluated using the death data of COVID-19 in Pakistan and Afghanistan. It has been verified that the EFEW model is capable of modeling both the monotonic and nonmonotonic failure data better than the existing models. Moreover, the findings consistently lead to better results and increase the model flexibility compared to the existing probability distributions. Hence, the inclusion of the parameter (*d*) to the existing model plays an important role and hence is a better choice in making predictions of deaths among infected patients of coronavirus than the other models.

It is expected that the present class of expressions, along with its special forms, will attract the researchers towards its contribution to other applied research areas such as engineering, hydrology, agriculture, economics, survival analysis, and various others. Moreover, the present study can be extended to neutrosophic statistics. A future research study may also be conducted on the Bayesian analysis of the model parameters under various loss functions.

## Figures and Tables

**Figure 1:** (a) Weekly average of COVID-19 infections in Pakistan. (b) Weekly average of COVID-19 infections in Afghanistan.

**Figure 2:** Plots of the CDF and PDF of EFEW.

**Figure 3:** Hazard rate function of EFEW.

**Figure 4:** Theoretical and empirical PDF and CDF of EFEW.

**Figure 5:** Theoretical, empirical, Q-Q plot, and P-P plot for EFEW.

**Figure 6:** TTT plot of the COVID-19 data.

**Figure 7:** Theoretical and empirical PDF and CDF of EFEW.

**Figure 8:** Theoretical, empirical, Q-Q plot, and P-P plot for EFEW.

**Figure 9:** TTT plot of the COVID-19 data of Afghanistan.

**Table 1:** Skewness and kurtosis.

*a*	*b*	*c*	*d*	Skewness	Kurtosis
0.5	9.5	0.1	1	0.996	43.031
0.5	10	10	10	0.010	1.239
15	15	15	0.1	-0.421	2.420
0.1	20	0.1	0.1	1	155
10	10	15	1	-0.017	1.254
10	7	4	1	0.009	1.251
1	10	1	10	0.123	1.277
1	10	0.1	0.1	0.999	121.275
10	10	10	0.1	-0.519	1.262
10	10	10	10	0.048	1.242

**Table 2:** Data set 1: Pakistan (total deaths per million).

0.009	0.014	0.014	0.023	0.027	0.032	0.036	0.041	0.05	0.054
0.063	0.095	0.118	0.122	0.154	0.181	0.186	0.213	0.24	0.258
0.276	0.294	0.299	0.389	0.412	0.421	0.435	0.503	0.579	0.611
0.647	0.761	0.797	0.91	0.96	1.073	1.145	1.218	1.272	1.322
1.412	1.553	1.743	1.888	1.992	2.069	2.155	2.327	2.553	2.648
2.712	2.879	2.983	3.196	3.336	3.445	3.486	3.776	3.776	3.952
4.088	4.251	4.459	4.604	4.83	4.984	5.129	5.283	5.419	5.546
5.704	5.962	6.315	6.714	6.985	7.338	7.642	8.013	8.321	8.76
9.063	9.358	9.833	10.209	10.666	11.15	11.15	11.549	12.354	12.852
13.468	14.002	14.618	15.311	15.849	16.252	16.728	16.999	17.669	17.936
18.267	18.643	18.864	19.485	19.897	20.25	20.603	20.603	20.911	21.558
21.907	22.282	22.559	22.898	23.192	23.527	23.84	24.084	24.383	24.564
24.564	24.999	25.207	25.347	25.528	25.7	25.845	26.09	26.198	26.357
26.357	26.447	26.551	26.674	26.818	26.941	26.941	27.054	27.158	27.158
27.226	27.321	27.398	27.47	27.534	27.602	27.67	27.747	27.792	27.855
27.896	27.955	27.955	28.023	28.073	28.109	28.154	28.208	28.267	28.267
28.317	28.371	28.403	28.444	28.448	28.466	28.494	28.512	28.647	28.679
28.702	28.702	28.724	28.747	28.788	28.815	28.838	28.851	28.878	28.896
28.924	28.942	28.969	29.01	29.041	29.046	29.064	29.082	29.118	29.141
29.173	29.204	29.231	29.272	29.308	29.331	29.354	29.422	29.458	29.485
29.485	29.53	29.585	29.625	29.662	29.689	29.743	29.788	29.824	29.883
29.942	29.974	30.051	30.123	30.146	30.209	30.295	30.341	30.399	30.454
30.494	30.508	30.535	30.599	30.671	30.762	30.811	30.888	30.943	31.006
31.088	31.205	31.341	31.432	31.545	31.586	31.69	31.785	31.939	32.106
32.183	32.328	32.414	32.563	32.731	32.812	34.229	34.419	34.687	34.841
35.058	35.325	35.506	35.75	35.954	36.149	36.33	36.629	36.968	37.145
37.394	37.588	37.851	38.019	38.421	38.693	38.947	39.173	39.494	39.82
39.983	40.314	40.789	41.106	41.486	41.876	42.238	42.518	42.89	43.265
43.768	44.153	44.438	44.701	44.95	45.235	45.484	45.746	46.068	46.439
46.679	46.855	47.123	47.358						

**Table 3:** Data set 2: Afghanistan (total deaths per million).

0.026	0.026	0.026	0.051	0.077	0.077	0.103	0.103	0.103	0.103
0.103	0.103	0.206	0.257	0.308	0.385	0.411	0.411	0.437	0.462
0.462	0.488	0.565	0.591	0.745	0.771	0.771	0.771	0.848	0.925
0.925	1.028	1.028	1.105	1.207	1.336	1.49	1.516	1.567	1.644
1.747	1.85	2.183	2.312	2.44	2.672	2.723	2.8	2.954	3.083
3.134	3.262	3.391	3.494	3.93	4.316	4.367	4.444	4.573	4.829
4.984	5.292	5.574	5.626	5.651	5.677	5.857	6.062	6.345	6.422
6.628	6.833	7.039	7.655	7.809	8.04	8.503	9.273	9.582	9.967
10.506	11.046	11.56	11.688	12.202	12.382	12.716	13.05	14.129	14.18
14.719	15.028	15.336	15.85	16.389	17.314	17.519	18.393	18.701	19.009
19.318	20.037	20.782	21.09	21.27	22.246	23.119	23.685	24.121	24.635
24.995	25.585	25.996	26.716	27.332	28.154	28.694	29.516	29.952	30.389
30.441	30.518	30.62	31.16	31.519	32.085	32.393	32.65	32.675	32.701
32.958	32.984	33.009	33.035	33.138	33.138	33.292	33.42	33.652	33.78
33.934	34.14	34.576	34.833	35.064	35.193	35.219	35.347	35.398	35.501
35.553	35.604	35.604	35.604	35.655	35.707	35.912	36.015	36.015	36.041
36.041	36.041	36.041	36.143	36.22	36.22	36.22	36.22	36.297	36.375
36.452	36.503	36.503	36.503	36.503	36.503	36.657	36.683	36.94	36.94
36.965	36.965	37.068	37.145	37.171	37.197	37.325	37.325	37.376	37.376
37.453	37.505	37.505	37.505	37.505	37.608	37.608	37.71	37.736	37.787
37.813	37.864	37.89	37.993	38.044	38.07	38.096	38.096	38.198	38.275
38.378	38.507	38.558	38.609	38.712	38.764	38.866	38.943	39.046	39.175
39.329	39.406	39.431	39.508	39.508	39.663	39.74	39.842	39.997	39.997
40.048	40.202	40.51	40.587	40.69	40.947	41.05	41.307	41.615	42
42.154	42.334	42.463	42.797	43.105	43.413	43.721	44.055	44.389	44.62
44.698	45.006	45.571	46.11	46.804	47.292	47.42	47.42	47.883	48.14
48.808	48.962	49.296	49.707	49.964	50.246	50.477	50.58	51.248	51.659
52.019	52.147	52.584	53.098	53.483	53.843	54.382	54.613	54.947	55.204
55.487	55.846	55.975	56.026	56.283	56.283	56.283	56.283	57.465	57.644

**Table 4:** MLE and standard errors for data 1.

Model	W	A	MLE	Standard error	-log(L)
EFEW	1.727	8.395	9.286	1.399	1090.112
			0.002	0.0002	
			1.886	0.0266	
			0.1901	0.0236	
FEW	4.284	22.263	1.989	0.3550	1187.638
			0.099	0.0239	
			0.882	0.0609	
Ex-W	4.711	24.596	3.834	NaN	1204.855
			0.999	NaN	
			-3.796	NaN	
W	4.679	24.424	0.042	0.0081	1203.33
			1.020	0.0543	
E	4.705	24.563	0.045	0.0026	1203.454
AIFW	2.756	13.822	0.019	0.0020	1229.493
			0.050	0.0026	
GAPW	4.339	22.566	0.362	0.0791	1190.373
			0.085	0.0180	
			0.908	0.0542	

**Table 5:** Model selection criterion for data 1.

Models	AIC	CAIC	BIC	HQIC
EFEW	2188.224	2188.362	2202.958	2194.124
FEW	2381.277	2381.359	2392.327	2385.702
E	2408.907	2408.921	2412.591	2410.383
W	2410.659	2410.701	2418.027	2413.61
Ex-W	2415.711	2415.794	2426.762	2420.136
AIFW	2462.986	2463.028	2470.354	2465.937
GAPW	2386.745	2386.828	2397.796	2391.171

**Table 6:** MLE and standard errors for data 2.

Model	W	A	MLE	Standard error	-log(L)
EFEW	1.792	8.989	7.784	1.1655	1155.904
			0.002	0.0002	
			1.775	0.0249	
			0.219	0.0263	
FEW	3.779	19.969	1.775	0.3369	1236.656
			0.072	0.0158	
			0.902	0.0517	
E	4.122	21.839	0.036	0.0021	1249.168
W	4.072	21.563	0.031	0.0071	1248.961
			1.043	0.0600	
Ex-W	4.063	21.519	3.137	NaN	1254.047
			0.999	NaN	
			-3.095	NaN	
AIFW	2.487	12.846	0.045	0.0049	1278.144
			0.042	0.0022	
GAPW	3.850	20.354	0.418	0.1003	1238.872
			0.068	0.0189	
			0.909	0.06515	

**Table 7:** Model selection criterion for data 2.

Models	AIC	CAIC	BIC	HQIC
EFEW	2319.808	2319.949	2334.488	2325.69
FEW	2479.313	2479.396	2490.322	2483.724
E	2500.336	2500.35	2504.006	2501.806
W	2501.923	2501.965	2509.263	2504.863
Ex-W	2514.095	2514.178	2525.104	2518.506
AIFW	2560.288	2560.33	2567.628	2563.228
GAPW	2483.744	2483.828	2494.754	2488.155

**Table 8:** Average values of MSE and bias.

Parameters	n	MSE (*a*)	MSE (*b*)	MSE (*c*)	MSE (*d*)	Bias (*a*)	Bias (*b*)	Bias (*c*)	Bias (*d*)
*a* = 0.5	40	31.947	5.718	1.119	48.202	3.904	1.907	0.949	5.032
*b* = 0.05	70	24.757	5.100	1.032	41.127	3.392	1.720	0.901	4.521
*c* = 1.5	100	22.843	4.316	0.918	34.410	3.280	1.498	0.833	3.829
*d* = 0.5	150	20.125	3.659	0.831	26.742	2.983	1.309	0.781	3.190
*a* = 0.6	100	21.828	3.174	1.090	30.497	3.034	1.210	0.888	3.450
*b* = 0.05	200	13.441	1.606	0.724	16.210	2.239	0.714	0.676	1.976
*c* = 1.77	300	9.5134	1.047	0.577	11.166	1.768	0.528	0.581	1.472
*d* = 0.6	400	7.8027	0.758	0.492	8.0283	1.558	0.425	0.513	1.140

## Data Availability

The simulated data used to support the findings of this study are included within the article.
